This article has been retracted.

# Legal Guarantee of Smart City Pilot and Green and Low-Carbon Development

**DOI:** 10.1155/2022/4280441

**Published:** 2022-09-26

**Authors:** Na Yan

**Affiliations:** Law School, Guangxi Normal University, Guilin 541001, Guangxi, China

## Abstract

Green and smart cities are based on clean energy and rely on information technology. They are the guarantee for the realization of efficient and intelligent urban development and green ecological transformation, the basis for sustainable social and economic development, and the inevitable trend of urban development. Therefore, the evaluation of the development level of green and smart cities is of great significance to the development of Chinese cities. This paper has aimed to study the issue of smart city pilots and legal guarantees for green and low-carbon development and introduced the concept of smart city line management, as well as the related theory of entropy weight method, cloud model, and support vector machine algorithm. Based on the sustainable development index system, this paper has combined the low-carbon concept to construct the low-carbon city evaluation index system and carried out an empirical analysis. The sustainable development index system, the research results of low-carbon city, and the current situation and characteristics of low-carbon city construction are studied and analyzed. On this premise, a low-carbon city assessment framework in view of reasonable improvement is built, including low-carbon economy, low-carbon society, low-carbon climate, and low-carbon component. The experimental results of this paper show that the low-carbon environment subsystem has the best coordinated development among the four subsystems, and the current state is the best. By 2021, the coordination degree value has reached 0.6656, which is in a relatively coordinated state.

## 1. Introduction

With the development of new technologies such as the huge amount of information, the Internet of Things, and distributed computing, the concept of metropolitan development has been continuously improved, and this is only the tip of the iceberg. The innovative concept of further development has been incorporated into the field of metropolitan development. A new impetus for urban development was provided. With the development of cities, smart cities gradually replace digital cities and become the highest stage of urban development. Since IBM introduced the term “smart planet” in 2008, more than 50 countries including the United States, Sweden, Japan, Singapore, and South Korea have begun to build smart city pilot projects. In fact, as of May 2016, more than 550 cities in 95% and 85% of the cities above the county level in China are building smart cities. This paper has traced the development process of smart cities, combined with the new planning and construction of sustainable urban development in the “13th Five-Year Plan.” From the investigation of green and brilliant urban communities, the assessment file arrangement of China's green and shrewd urban communities is laid out, the advancement level of China's green and savvy urban communities is all the more precisely assessed, and the local distinctions of China's green and brilliant urban areas and the explanations behind the distinctions broke down. It is convenient to draw relevant advanced experience from it, so as to accurately locate different regions of China. It can find solutions to problems and improve strategies for builders to grasp the direction of urban development. It will provide new impetus for the sustainable development of cities and provide certain support for improving the level of China's green and smart construction. The innovation of this paper is that exploring the connotation and goals of green smart city can enrich the relevant theories and research methods of green smart city and expand the research horizon.

## 2. Related Work

With the improvement of society, individuals give increasingly more consideration to low-carbon ecological security. To decrease creation cost and acknowledge green creation process, Guo et al. proposed a new method for preparing activated carbon by ammoniation activation method to improve its physicochemical properties and adsorption properties [1]. Qu et al. synthesized a porous silicon-carbon composite extracted from paper mill sludge and used for rapid iodine capture [2]. Chu et al. investigated two cases to upgrade the water center into a “green gas station” for a low-carbon city. Green gas stations include biomethane, green hydrogen supply systems, and power supply systems [3]. Holm and Vennervirta concentrated on how professional schooling and preparing and advanced education could add to a green and low-carbon economy in Finland [4]. In any case, the deficiencies of these examinations are that the model development is not logical and sufficiently sensible. The information actually should be taken to the next level.

With the advancement and innovation of science and technology, the support vector machine algorithm has penetrated into all aspects of personal life. This is just the beginning, and more and more researchers are working on it. The combination of the microfluidic sensor proposed by Jinhong and the support vector machine algorithm provides a promising platform for the construction of sensor networks in smart hospitals [5]. Aiming at the operation status of medium and low-pressure gas regulators in SCADA systems, Hao proposed a new safety precaution method for gas regulators based on support vector machine (SVM) [6]. Shyamala et al. proposed a SVM-based damage detection strategy, which is performed step-by-step by first locating and then determining the severity of the damage [7]. Zhu talked about the ongoing models of energy oversight frameworks at home and abroad, worked on the strategy in blend with the deficiencies of information mining, and afterward applied the help vector machine (SVM) calculation to the web-based business energy oversight model [8]. The drawback of these examinations, in any case, is that the contemplations are not adequately extensive to adjust to additional perplexing circumstances, and accuracy should be moved along.

## 3. Relevant Methods for Smart City Pilots and Legal Guarantees for Green and Low-Carbon Development

### 3.1. Smart City

#### 3.1.1. Theoretical Framework of Smart City

The concept of smart city is built on the basis of digital city, which digitizes information in different fields and geographical locations such as economy, culture, and transportation. The smart city has added a perception layer composed of technical terminal equipment such as radio frequency identification and infrared induction. Data collection is carried out, and the processing work after the collected data is formed through the huge Internet of Things data connection and sharing. Finally, through the analysis of data information, various applications based on data platforms are optimized. Among them, the Internet of Things, cloud computing, and big data technologies are widely used in all aspects of smart city construction, making urban development more intelligent (Figure 1) [9, 10].

#### 3.1.2. Construction of the Evaluation Index System

*(1) Theoretical Connection of Secondary Indicators*. The core composition of a city is people, and it is also the result of the agglomeration effect of people, and smart cities also aim to improve the efficiency between people in urban space. The regular life of people in cities divides individual people into three major organizational groups. First, government organizations are responsible for rational planning and management of basic urban public services. The second is enterprise organization, which forms the basic commercial activities of the city. Finally, there are thousands of family groups in the city, and it is also the most basic activity group in the city. The core of a smart city is how to use the Internet of Things, cloud computing, big data, and other network components to improve the efficiency of the relationship between the government, enterprises, and individuals [11]. Therefore, from the perspectives of the government, enterprises, and individuals, three indicators representing smart cities can be summarized, namely, smart city online government, smart city industrial economy, and smart city humanistic environment. On this basis, the strengthening of the connection between the three requires a basic network. Therefore, it needs to add the indicator of smart city infrastructure, and finally whether it is a government organization or a business organization. From the perspective of an individual person, one needs to live, to travel, to see a doctor, to travel, and so on. Therefore, a smart city life service indicator is added at the end.

As shown in Figure 2, under the mesh envelope of smart city infrastructure and life services, the efficiency of the connection between the government, enterprises, and people is improved, making the city more intelligent.

*(2) Evaluation Index System*. The scientific, practical, operable, and guiding principles are the core of the evaluation index system. The existing literature on the smart city indicator system is complex and diverse, but considering the completeness and availability of statistical data in various cities in Hebei Province, indicators such as the level of democracy and environmental awareness are not used as evaluation indicators in this paper. This paper extracts the statistical indicators related to the construction of smart cities by sorting out the existing indicators and searching according to the China Urban Statistical Yearbook and Internet data [12, 13]. The selection of indicators covers the most basic smart city basic indicators such as transportation, medical care, tourism, education, technology, entertainment, and life. The most basic indicators are obtained in two categories: one is obtained from the Urban Statistical Yearbook, and the other is obtained from Internet search data. And the basic data are classified and merged with weights, and the index system is sorted out, as shown in Table 1.

There are a total of 12 three-level indicators, which are obtained through basic data. Smart city infrastructure is measured by mobile phones, internet broadband, and the distribution of the three major operators. The smart city industrial economy is represented by industry, network economy, and innovation. Smart city online government is represented by online and online information release. Smart city life services are represented by network applications such as transportation, medical care, and tourism, and online processing of life services. Finally, the humanistic environment of the smart city is represented by the education situation of people and the urban environment where people live [14].

#### 3.1.3. The Main Body of Green Smart City

The main body of green smart city includes almost all social organizations and individuals; specifically, it can be divided into the government, enterprises, and citizens.

*(1) Government*. The government plays the role of “brain” in the city, and its importance determines that the core task of building a green smart city is to build a smart government. The government can organize regulation through policy guidance, strategic planning, and regulatory constraints. Therefore, it will play a guiding role in the development of China's green and smart cities [15]. The top-level design of a green smart city can be planned. From the perspective of a leader, the overall structure of the smart city can be comprehensively designed, and all aspects of the overall structure can be planned. Reasonable top-level design and overall planning blueprint are conducive to resource sharing between cities, industries, and departments [16]. It is helpful to clarify the development direction of the city. It is beneficial to improve resource utilization by supporting the development of science and technology. In the “Internet +” era, the Chinese government's administrative system has entered a period of deepening transformation and reform. Under the new normal, smart government has gradually replaced e-government and has become an advanced stage of e-government development. Smart government is centered on big data analysis and supported by modern information technology. Information resources are screened, optimized, and reorganized. The smart government cloud platform is built to implement data exchange and resource sharing, thereby saving government costs. Transparency and fairness in government affairs are increased. The work efficiency and decision-making ability of government management services are improved [17].

*(2) Enterprise*. In urban construction, the role of enterprise development is far greater than that of the government. The government is the guide, and the enterprise is the leading [18]. Enterprises are the main body of the market economy. In the market, there are not only public service products provided by the government, but also products that conform to the rules of market competition. The main role of enterprises in the construction of green and smart cities is to implement the development of related industries and promote the application of related industries and products in various fields.

*(3) Residents*. The ultimate goal of building a green and smart city is to serve people and enable urban residents to live a better life. The government needs to encourage more enterprises and residents to actively participate in it. Occupants are both makers and buyers in the development of green and shrewd urban communities. Occupants accept various jobs and partake in the whole course of metropolitan development. The public authority can work on occupants' attention to natural security and the capacity to take part in the development of green and brilliant urban communities through exposure, advancement, schooling, and preparing connected with green and savvy urban areas. Residents are encouraged to participate in construction, and the values of harmonious coexistence and common development between man and nature and the concept of green consumption are advocated; residents' participation is fully utilized, natural resources and information resources are optimally allocated, and the construction of green and smart cities is supervised and promoted.

### 3.2. Theories Related to the Entropy Weight Method

#### 3.2.1. Overview of the Entropy Weight Method

Entropy was initially only an idea of thermodynamics in material science and, later, brought into data hypothesis, called “information entropy,” which has been widely used in various engineering or economic fields [19, 20]. The entropy weight method is an objective method for determining weights, which has the characteristics of wide applicability, high accuracy, and strong objectivity. The basic idea of the entropy weight method is to determine the weight of each indicator according to the degree of variation of each variable and then modify it to obtain a relatively objective weight [21, 22]. The entropy weight method has a strong mathematical theoretical basis and can objectively and accurately determine the index weight, avoiding the influence of subjective factors of other subjective weighting methods.

#### 3.2.2. Determining the Weight by the Inheritance Law

Let the initial data matrix of object set A be

(1) $$\begin{array}{c} A={\left(a_{ij}\right)}_{n\times m}. \end{array}$$

It includes *n* objects to be evaluated and *m* evaluation indicators.

Then, the detailed steps to obtain the evaluation index weight by using the direct right method are as follows.

**Step 1 .**

Standardize the initial indicator data: set the normalized value of each indicator data, and then, there are

(2) $$\begin{array}{c} B_{ij}=\frac{A_{ij}-\min\left(A_{i}\right)}{\max\left(A_{i}\right)-\min\left(A_{i}\right)}. \end{array}$$

**Step 2 .**

Calculate the data relative worth of each record: the data relative worth of the jth gathering of file information is

(3) $$\begin{array}{c} Q_{j}=-\ln\;{\left(n\right)}^{-1}\sum_{k_{ij}}^{n}\ln\;k_{ij},\\ k_{ij}=\frac{B_{ij}}{\sum_{i=1}^{n}B_{ij}}. \end{array}$$

If

(4) $$\begin{array}{c} k_{ij}=0, \end{array}$$

then define

(5) $$\begin{array}{c} \underset{k_{ij}⟶0}{\lim}k_{ij}\ln\;k_{ij}=0. \end{array}$$

**Step 3 .**

Calculate the indicator weight vector:

(6) $$\begin{array}{c} \omega =\left\{\omega_{1},\omega_{2},\ldots ,\omega_{n}\right\},\\ \omega_{j}=\frac{1-Q_{j}}{\sum_{j=1}^{m}\left(1-Q_{j}\right)},\\ 0\leq \omega_{j}\leq 1,\\ \sum_{j=1}^{m}\omega_{j}=1. \end{array}$$

### 3.3. Theories Related to Cloud Models

This paper evaluates the development level of green and smart cities, and there will inevitably be certain uncertainties. Therefore, in order to make a reasonable and effective evaluation, the inevitability of the existence of uncertain factors should be noticed. To address the unavoidable uncertainty, other evaluation methods are compared. This paper finally chooses to use the direct right method-cloud model to evaluate the development level of China's green and smart cities.

#### 3.3.1. The Concept of the Cloud Model

Natural language is the crystallization of human wisdom and the carrier of knowledge, but natural language contains too much uncertainty. To study the expressions and methods of uncertainty in language, it is necessary to establish a qualitative and quantitative mutual conversion model, as the basis for the transformation of natural language and data language.

Let *M* be a quantitative universe, and let *C* be a qualitative concept on the quantitative universe M, and the quantitative value a is a random realization of C, that is, *a* ∈ *M*, and the random number *μ*(*a*) is the degree of certainty that a realizes on C, *μ*(*a*) ∈ [0,1], and has Stable Tendency:

(7) $$\begin{array}{c} \mu \left(a\right):M⟶\left[0,1\right],\\ \forall a\in M,\\ a⟶\mu \left(a\right). \end{array}$$

Then, the distribution of a on the universe of discourse M is called a cloud, and the random number reflects the degree of certainty of the quantitative value a to the qualitative concept C.

#### 3.3.2. Digital Features of Cloud Models

The overall characterization of the cloud model concept can be used to represent the mathematical properties of linguistic values by using the cloud's numerical features—expectation (*E*_*a*_), entropy (*E*_*n*_), and hyperentropy (He) [23, 24]. Expectation *E*_*a*_: the point where cloud droplets are reflected in domain M that best represents qualitative concepts. Entropy *E*_*n*_ : the probability and ambiguity of qualitative concepts are represented, which can reflect not only the discrete degree of cloud droplets, but also the value range of cloud droplets. Hyperentropy He: the entropy of entropy, representing the uncertainty measure of entropy. Taking (0, 1, 0.1) as the three digital features of the cloud model and 5000 cloud droplets as an example, the one-dimensional normal cloud model is shown in Figure 3.

### 3.4. Support Vector Machines

#### 3.4.1. The Concept of Support Vector Machine

Support Vector Machine (SVM) identifies the evaluation object by constructing the optimal decision hyperplane, so as to transform the optimization problem into the relevant classification and regression analysis problems to obtain the optimal results [25]. It is based on the VC dimension theory (Vapnik–Chervonenkis Dimension) in statistical theory and the principle of minimum structural risk.

The specific idea of SVM to solve the problem is reflected in two aspects: one is to classify the linearly separable evaluation objects. The second is to develop the ideal order hyperplane by applying the guideline of limiting primary gamble in the low-layered example space, to get the ideal outcome (Figure 4).

#### 3.4.2. Regression Prediction Algorithm of Support Vector Machine

From the perspective of support vector machine regression prediction used in this paper, considering that the main algorithms used in support vector regression prediction are the algorithms of insensitive function and kernel function, the specific algorithms are summarized as follows:

*(1) SVM Regression Prediction Algorithm*. Let sample set

(8) $$\begin{array}{c} X=\left\{\left(b_{l},a_{l}\right)|b_{l}\in R,a_{l}\in R^{\text{d}}\right\}. \end{array}$$

The regression function is expressed linearly as

(9) $$\begin{array}{c} g\left(a\right)=\omega^{T}\phi \left(a\right)+y. \end{array}$$

In order to minimize the structural risk of the regression function *g*(*a*), that is, to achieve min1/2*ω*^*T*^*ω*, it is necessary to seek *ω* and *b*. The optimal regression function can be determined by the minimum value of the function, and the nonnegative slack variable *ξ*_*i*_ and the penalty factor C are introduced to obtain

(10) $$\begin{array}{c} \min\left(\frac{1}{2}\omega^{T}\omega +C\sum_{i=1}^{l}\left(\xi_{i}+\xi_{i}^{*}\right)\right), \end{array}$$

where *ω* represents the dimension, C is a constant that has been determined, and slack variables control the upper and lower bounds of the output constraints.

(11) $$\begin{array}{c} \left\{\begin{array}{c} b-\omega^{T}\phi \left(a_{i}\right)-y\leq \varepsilon +\xi_{i},\\ \omega^{T}\phi \left(a_{i}\right)+y-b\leq \varepsilon +\xi_{i}^{*},\\ \xi_{i},\xi_{i}^{*}\geq 0. \end{array}\right. \end{array}$$

Introduce the Lagrange multiplier:

(12) $$\begin{array}{c} L=\frac{1}{2}\omega^{T}\omega +C\sum_{i=1}^{l}\left(\xi_{i}+\xi_{i}^{*}\right)-\sum_{i=1}^{l}\left(\varepsilon +\xi_{i}-b+\left(\omega^{T}\phi \left(a_{i}\right)\right)+y\right),\\ -\sum_{i=1}^{l}\alpha_{i}\left(\varepsilon +\xi_{i}+b-\left(\omega^{T}\phi \left(a_{i}\right)\right)-y\right)-\sum_{i=1}^{l}\left(\eta_{i}\xi_{i}+\eta_{i}^{*}\xi_{i}^{*}\right). \end{array}$$

In the formula, *α*_*i*_ is the Lagrangian product factor. If the non-zero factor in the multiplication factor *α*_*i*_ is represented by *α*_*i*_^0^, then *α*_*i*_^0^ is the support vector obtained through training by using support vector machine (SVM) [26].

*(2) Kernel Function*. Kernel functions play an important role in SVM operations, not only to solve the nonlinear latitude problem, but also to replace the direct inner product operation in the high-dimensional feature space. There is no need to specify the function of a certain high-dimensional space, and the high-dimensional operation is simplified [4, 27].

For building choice guidelines, three normal sorts of SVMs are given as follows:

(1) Polynomial machine with part capability:
  (13) $$\begin{array}{c} D\left(h,h_{i}\right)={\left(h•h_{i}+1\right)}^{r}, \end{array}$$
where *r* is the request for the polynomial piece.
(2) Radial premise capability machine with piece capability:
  (14) $$\begin{array}{c} D\left(h,h_{i}\right)=\exp\left(\frac{-1}{\delta^{2}{\left(h-h_{i}\right)}^{2}}\right), \end{array}$$
where *δ* is the bandwidth of the radial basis function kernel.
(3) Two-layer brain network machine with piece capability:
  (15) $$\begin{array}{c} D\left(h,h_{i}\right)=F\left[\left(h•h_{i}\right)\right],\\ =\frac{1}{1+\exp\left(v\left(h•h_{i}\right)-b\right)}, \end{array}$$
*v* and *b* are the parameters of the F-shaped function *F*[(*h*•*h*_*i*_)] satisfying the inequality *b* ≥ *v*.

The basic idea of SVM is shown in Figure 5.

## 4. Experiments on Legal Guarantees for Smart City Pilots and Green and Low-Carbon Development

After the low-carbon city development document framework is formulated, it should be utilized and the practicability and feasibility of the filing framework should be tested. Considering that Shanghai is one of the principal pilot low-carbon urban communities in China, and the information measurements are moderately finished and simple to get, Shanghai is picked for instance. The utilization of this file framework and the reception of sensible assessment techniques do a particular assessment that concentrates on the development of low-carbon city in Shanghai. It gets the improvement of the city, in this manner, giving a reference to future turn of events.

As China's monetary, exchange, show, and delivery focus, Shanghai focuses closer on feasible improvement, while the economy is growing quickly. As one of the main pilots of a low-carbon city, Shanghai has gone all out in the development of a low-carbon city and has accomplished productive outcomes; however, there are as yet numerous issues and colossal difficulties.

Doing the act of metropolitan low-carbon life in Shanghai, the principal items in the task plan include the following: first and foremost, to research the energy utilization of structures and further develop the energy proficiency of huge structures. The World Wide Fund for Nature collaborated with the Shanghai Institute of Building Research and the Shanghai Construction and Transportation Commission to carry out the work and selected large commercial buildings such as shopping malls, office buildings, and hotels as pilot projects. The energy consumption of these buildings is investigated, calculated, and made public. The second is to start the training of building industry managers. The energy-saving operation capability of the building will be improved by training relevant management personnel. The third is the policy research on ecological building development and the selection and implementation of demonstration projects.

### 4.1. Evaluation Index Data Collection

As indicated by the built low-carbon city assessment file framework, the assessment of low-carbon city development and advancement incorporates four subsystems: low-carbon economy (A1), low-carbon society (A2), low-carbon climate (A3), and low-carbon system (A4). There are specific evaluation indicators under different subsystems. There are 13 specific indicators. It chiefly remembers the extent of tertiary industry for GDP (A11), energy utilization per unit of GDP (A12), energy utilization per unit of modern added esteem (A13), per capita energy utilization (A21), utilization of public vehicle vehicles per 10,000 individuals (A22), urban per capita lodging living region (A23), modern wastewater release consistence rate (A31), metropolitan sewage treatment rate (A32), per capita green region (A33), air quality magnificent rate (A34), fossil fuel byproducts (A35), R&D as a level of monetary consumption (A41), and Internet client infiltration rate (A42). The concept of “low-carbon economy” was formally proposed in 2003, and it has been widely concerned and developed in various countries. In addition, according to the availability of data, the selection and collection of evaluation index data began in 2017. The Shanghai Statistical Yearbook over the years was searched, and the specific data of Shanghai evaluation indicators from 2017 to 2021 were collected as shown in Table 2.

Sorting is carried out by performing fuzzy operations on the judgment matrix of the above subsystems and specific indicators under the subsystems. The final weights of indicators at all levels are shown in Table 3.

### 4.2. Coordination Degree Model

To calculate the coordination degree, the efficacy value of each evaluation index in the system must be calculated first. According to the formula of the efficacy function, the upper and lower limit values of the indicators at the critical point of system stability need to be determined. Since the concept of “low-carbon economy” was formally proposed in 2003, the concept of low-carbon was paid attention to and applied in practice after that. In addition, considering that low-carbon-related indicators began to be counted in 2004. Therefore, the data in 2004 is used as the lower limit. The selection of the upper limit value is generally a future development goal. Therefore, the upper limit is the development goal to 2015 proposed in Shanghai's “Twelfth Five-Year Plan.” For those that are not clearly specified in the “Twelfth Five-Year Plan,” the trend extrapolation method is used to forecast, and the forecast value is taken as the upper limit. The upper and lower limits of the specific indicators in each subsystem are shown in Table 4.

The collected current value of each evaluation index in Shanghai and the above-determined upper and lower limit values are brought into the function formula, and also, every subsystem in the assessment file arrangement of Shanghai's low-carbon city development from 2017 to 2021 is gotten. The viability upsides of the assessment markers are displayed in Figure 6.

### 4.3. Evaluation Results

The low-carbon city construction in Shanghai from 2017 to 2021 was evaluated using the coordination degree model based on triangular fuzzy hierarchy. The development status of the system and the overall coordination degree of the main components between the systems can be seen from the final coordination degree value:

1. Overall, the overall coordination degree of Shanghai has been developing towards a high degree of coordination. The specific change trend is shown in Figure 7. As can be seen from the figure, in 2017, the total coordination degree was 0.1509, which was in a very uncoordinated state. After that, the total coordination degree generally showed an upward trend, especially by 2020, and the total coordination degree was 0.5015. For the first time, the basic coordination state is reached. This is closely related to the fact that Shanghai was listed as a low-carbon city pilot in 2019 and began to pay more attention to the development of low-carbon cities. By 2021, the overall coordination degree of Shanghai's low-carbon city development will be 0.5675, which has achieved greater development compared with 2020 and is approaching a more coordinated state. This shows that the overall development of Shanghai's low-carbon city construction is relatively rapid.
2. From the subsystem level, the four subsystems of Shanghai's low-carbon economy, low-carbon society, low-carbon environment, and low-carbon mechanism show a continuous development trend from an overall perspective. The specific trends are shown in Figure 8.
3. It can be seen from Figure 8 that the coordination degree of the low-carbon economy has risen rapidly, showing a linear upward trend. In just 5 years from 2017 to 2021, the coordination degree value has risen from 0.0379 to 0.5983, which is close to a relatively coordinated state. This shows that Shanghai is paying more and more attention to low carbon while achieving rapid economic growth. The coordination degree of the low-carbon society is poor, and it will still be in a state of disharmony by 2021, and the coordination degree value will be negative in 2019 and 2020. This is because the specific indicator value of public vehicles owned by every 10,000 people in this subsystem has dropped sharply in the past two years, resulting in unreasonable coordination value. The low-carbon environment subsystem has the best coordinated development among the four subsystems, and the current state is the best. By 2021, the coordination degree value has reached 0.6656, which is in a relatively coordinated state, indicating that Shanghai is in a state of environmental protection, especially reducing carbon emissions. Extraordinary headway has been made in ecological assurance. The coordination degree worth of the low-carbon component has developed consistently, coming to 0.6074 by 2021, and a moderately planned state has likewise been accomplished, mirroring that Shanghai connects incredible significance to the improvement of low-carbon economy and low-carbon urban communities and has given more prominent help and exposure. In general, in these four subsystems, the low-carbon climate and low-carbon components are in a somewhat organized state and are well nurtured, while the low-carbon economy and low-carbon society are still in the basic planning state and should be further developed.
4. Based on the particular assessment pointers under every subsystem, under the low-carbon economy, the energy utilization per 10,000 yuan of GDP and the energy utilization per unit of modern added esteem have arrived at a somewhat planned state. The proportion of the tertiary industry in GDP is still in an uncoordinated state: in a low-carbon society, the per capita living area in urban areas has reached a highly coordinated state, while the coordination between per capita energy consumption and public vehicles per 10,000 people is low. In a low-carbon environment, except that the discharge compliance rate of industrial wastewater is still in an uncoordinated state, other indicators are relatively coordinated. Under the low-carbon mechanism, the penetration rate of Internet users has achieved a high degree of coordination, while the ratio of R&D to fiscal expenditure is not in a coordinated state. It shows that the government should continue to increase investment in the construction of low-carbon cities.

## 5. Conclusions

Green development is a change from the past development model, and it is based on the tolerance of the environment and the limited use of resources, taking ecological protection as a critical reference in China's development. In addition, the continuous breakthrough of China's economy often leads to damage to the ecological balance and waste of resources. In order to minimize its negative impact, green development is an inevitable choice. This article discusses the issue of circular economy legal safeguard mechanism at this level, mainly using interdisciplinary and empirical research methods to conduct in-depth research on China's relevant legislation, law enforcement, judiciary, and law-abiding safeguard mechanisms. Then, from the three aspects of government promotion mechanism, market adjustment mechanism, and public participation mechanism, a circular economy legal guarantee mechanism for China's green development is constructed, so as to find a green and ecological development path with Chinese characteristics.

With the progressive exhaustion of worldwide energy and the persistent extending of the idea of feasible turn of events, people started to look for new improvement strategies, and the idea of low-carbon economy and low-carbon city appeared. Low-carbon economy and low-carbon city complement each other. The development of a low-carbon city requires a low-carbon economy as the foundation, and the development of a low-carbon economy requires a low-carbon city as a backing. China has gradually settled in Shanghai, Baoding, and other low-carbon pilot cities to explore the improvement model of low-carbon urban communities. The development of a low-carbon city is a course of persistent investigation, and a sensible assessment of the improvement status of a low-carbon city has turned into a vital connection in this cycle. It can give dynamic premise to the further improvement of low-carbon urban communities and advance the advancement of low-carbon urban communities in a superior bearing. Accordingly, the examination on the assessment of low-carbon city development is of incredible importance. Based on concentrating on the practical advancement record framework and low-carbon meaning, this paper has developed the low-carbon city assessment file framework and presented the three-sided fluffy number insightful pecking order process and the coordination degree model to build the fluffy coordination degree model for the development of low-carbon urban areas. Finally, Shanghai is regarded as a model of low-carbon city development and a pilot project for low-carbon city evaluation.

## Figures and Tables

**Figure 1:** The theoretical framework of smart cities.

**Figure 2:** Smart city secondary finger connections.

**Figure 3:** One-dimensional normal cloud map formed by 5000 cloud droplets with (0, 1, 0.1) as eigenvalues.

**Figure 4:** Schematic diagram of the structure of the support vector machine.

**Figure 5:** Basic idea of support vector machine.

**Figure 6:** 2017–2021 low-carbon economy subsystem indicator efficacy values.

**Figure 7:** The overall coordination trend of low-carbon city development in Shanghai from 2017 to 2021.

**Figure 8:** The trend of coordination degree of various subsystems of low-carbon city evaluation in Shanghai from 2017 to 2021.

**Table 1:** Smart city evaluation index system.

Primary index	Secondary indicators	Tertiary indicators
Smart city	Smart city infrastructure	Mobile phone index
		Internet broadband index
		Operator distribution index
	Smart city industrial economy	Smart industry development index
		Network economy development index
		Innovation development index
	Smart city online government	Online government index
		Information release index
	Smart city life service	Intelligent application index
		Smart convenience index
	Cultural environment of smart city	Education index
		Environmental index

**Table 2:** Historical data of evaluation indicators.

Index	2017	2018	2019	2020	2021
A11 (%)	52.2	54.5	55.99	59.37	57.4
A12 (tons of standard coal/10000 yuan)	0.861	0.804	0.774	0.728	0.713
A13 (ten thousand yuan per ton of standard coal)	1.188	1.126	1.07	1.028	0.953
A21 (tons of standard coal/10000 yuan)	4.520	4.685	4.768	4.692	4.848
A22 (vehicle/10000 persons)	12.64	12.30	10.62	11.09	12.45
A23 (*m*^3^)	16	16.5	16.9	17.2	17.6
A31 (%)	0.697	0.674	0.783	0.745	0.763
A32 (*m*^3^)	11.6	12.01	12.51	12.9	13
A33 (%)	37.2	37.6	38	38.2	38.1
A34 (%)	88.4	89.9	89.5	91.6	92.2
A35 (ten thousand tons/hundred million yuan)	2.092	1.93	1.809	1.719	1.622
A41 (%)	5.21	4.9	4.6	7.2	6.1
A42 (%)	52.8	58.1	61.4	65.1	68.1

**Table 3:** Weights in the low-carbon city evaluation index system.

Subsystem layer	Weight	Index layer	Weight
Low carbon economy (A1)	0.261	Proportion of tertiary industry I in GDP (A11)	0.233
		Energy consumption per 10000 yuan GDP (A12)	0.296
		Energy consumption per unit industrial added value (A13)	0.470
		Per capita energy consumption (A21)	0.446

Low carbon society (A2)	0.182	Use of public transport vehicles per 10000 people (A22)	0.350
		Urban per capita housing area (A23)	0.207
		Standard rate of industrial wastewater discharge (A31)	0.240
		Urban sewage treatment rate (A32)	0.171

Low carbon environment (A3)	0.420	Per capita green area (A33)	0.063
		Air quality excellence rate (A34)	0.145
		Carbon emissions (A35)	0.382

Low carbon mechanism (A4)	0.133	Ratio of R & D to fiscal expenditure (A41)	0.585
		Internet penetration rate of Sichuan households (A42)	0.415

**Table 4:** Upper and lower limits of specific indicators.

Index		Upper limit value	Lower limit value
Low carbon economy (A1)	A11 (%)	65.00	50.74
	A12 (lots of standard coal/10000 yuan)	0.598	0.916
	A13 (lots of standard coal/10000 yuan)	0.781	1.260
	A21 (lots of standard coal/10000 yuan)	5.838	4.041

Low carbon society (A2)	A22 (vehicle/10000 persons)	15	13.04
	A23 (m*'*)	18	14.799
	A31 (%)	85	0.494
	A32 (m3)	13.5	10.12

Low carbon environment (A3)	A33 (%)	38.5	36.000
	A34 (%)	95.000	85.1
	A35 (ten thousand tons/hundred million yuan)	1.344	2.286

Low carbon mechanism (A4)	A41 (%)	10.000	2.800
	A42 (%)	70.000	37.000

## Data Availability

This article does not cover data research. No data were used to support this study.
